The article "Direct Effects of Microalgae and Protists on Herring (Clupea harengus) Yolk Sac Larvae" was published in 2015. Journal: PLoS One.

# Direct Effects of Microalgae and Protists on Herring (*Clupea harengus*) Yolk Sac Larvae

**DOI:** 10.1371/journal.pone.0129344

**Published:** 2015-06-02

**Authors:** Björn Illing, Marta Moyano, Jan Niemax, Myron A. Peck

**Affiliations:** Institute of Hydrobiology and Fisheries Science, University of Hamburg, Olbersweg 24, Hamburg, Germany; Institut Maurice-Lamontagne, CANADA

## Abstract

This study investigated effects of microalgae (*Rhodomonas baltica*) and heterotrophic protists (*Oxyrrhis marina*) on the daily growth, activity, condition and feeding success of Atlantic herring (*Clupea harengus*) larvae from hatch, through the end of the endogenous (yolk sac) period. Yolk sac larvae were reared in the presence and absence of microplankton and, each day, groups of larvae were provided access to copepods. Larvae reared with microalgae and protists exhibited precocious (2 days earlier) and ≥ 60% increased feeding incidence on copepods compared to larvae reared in only seawater (SW). In the absence and presence of microalgae and protists, life span and growth trajectories of yolk sac larvae were similar and digestive enzyme activity (trypsin) and nutritional condition (RNA-DNA ratio) markedly declined in all larvae directly after yolk sac depletion. Thus, microplankton promoted early feeding but was not sufficient to alter life span and growth during the yolk sac phase. Given the importance of early feeding, field programs should place greater emphasis on the protozooplankton-ichthyoplankton link to better understand match-mismatch dynamics and bottom-up drivers of year class success in marine fish.

## Introduction

For nearly a century, fisheries scientists have been trying to gain a firm understanding of the processes affecting larval fish growth and survival, particularly during first feeding—a period that can act as a bottleneck for larval survival [1,2]. Besides abiotic factors (e.g. temperature, hydrography), the spatiotemporal overlap with predators and prey is assumed to be the strongest selection pressure affecting the survival of the offspring of marine fish species [3,4]. According to Houde’s ‘Stage Duration’ hypothesis [5], early and intense feeding is favorable since fast-growing individuals pass more rapidly through early stages most vulnerable to predation mortality and, in some years, fast growing larvae have a greater chance of survival than slower growers [6]. The potential for fast growth of marine fish larvae depends on a match in time and space between autotrophs and related blooms of zooplankton [7–9]. Marine fish larvae have poor energy reserves and a mismatch with their prey (traditionally considered to be various copepod species / stages) will soon cause them to pass the ‘point of no return’ [10], when poorly fed larvae are too weak to survive even if suitable prey becomes available.

In marine fish larviculture, microalgae and/or protists (‘green water’) are thought to increase the visual contrast of prey [11] helping young larvae forage more effectively, supply nutrients [12,13], help establish gut microbial flora by affecting bacterial populations in rearing water [14,15], and stimulate the appetite and production of digestive enzymes [16–18]. Furthermore, microalgae and protists may form a considerable portion of the gut contents of young larvae in nature [19,20]. However, few laboratory studies have examined this protozooplankton-ichthyoplankton link in detail and none, to the best knowledge, have examining the potential direct effects of microplankton at both the biochemical and organismal levels [6].

In this study we tested whether the passive ingestion of microalgae (*Rhodomonas baltica*) and heterotrophic protists (*Oxyrrhis marina*) by yolk sac larvae of southwest Baltic herring (*Clupea harengus*) would improve the success of early foraging of larvae on their preferred prey (nauplii of copepods [21]). Furthermore, we tested whether phytoplankton and protists benefitted larvae by extending the time between yolk-sac depletion and the ‘point of no return’, defined here as the time when larvae are too weak to feeding on copepods. In the southwest Baltic, the year class success of herring appears established during the larval (< 20 mm) phase [22] and successful first feeding by yolk sac larvae is one potential bottleneck to survival. The present study constitutes the first integrative (organismal- and biochemical-level) approach to explore the direct effects of microalgae and protists on the growth, development and aspects of nutritional fitness of marine fish yolk sac larvae.

## Material and Methods

### Ethical statement

All procedures involving animals were conducted in accordance with the German law on experimental animals and were approved by the responsible Ethical Committee of the department for food safety and veterinary matters which is part of the Hamburg Authority for Health and Consumer Protection (application nr. 95/11). Efforts were made to minimize suffering. For obtaining adult herring, no special permission was required since they were offered for sale by a commercial fisherman.

### Artificial spawning and egg incubation

Adult herring from the southwest Baltic Sea were caught using gillnets on 10^th^ April 2012 in Kiel Bight by a commercial fisherman (Northern Germany; 54.36°N, 10.16°E) and transferred on ice to the University of Hamburg. Two hours later, the eggs from 17 females were fertilized using the milt from 12 males at 9.3°C and a salinity of 15.0. The large number of parents was used to avoid the influence of maternal effects on offspring characteristics. The mean (±SD) standard length (*SL*) and wet weight of females were 23.0 (±1.5) cm and 141.6 (±25.1) g, and males were 23.3 (±1.2) cm and 163.0 (±32.2) g. Developing eggs were transferred to 90-l tanks within a temperature-controlled room and incubated at 9.9±0.2°C and a salinity of 16.0±0.4 (mean±SD). All tanks (used here and in experiments) were semi-static with 50% water replacements d^-1^ of filtered sea water (0.5 μm, Reiser Filtertechnik GmbH, Seligenstadt am Main), had gentle aeration and a light regime of 14:10 (L:D) was used. The embryos synchronously hatched at 13 days post-fertilization.

### Experimental Design and Sampling

Within ca. 10 h of hatch, yolk sac larvae were randomly attributed to one of two treatments and carefully transferred to experimental dark-green 50-l tanks with 3 replicate tanks per treatment (1200 larvae per tank). The two treatments consisted either of only seawater (SW) or SW with a combination of the cryptophycean algae *Rhodomonas baltica* (RB, 10,000 cells ml^-1^ = 540 μg C l^-1^) and the heterotrophic dinoflagellate *Oxyrrhis marina* (OX, 1,000 cells ml^-1^ = 196 μg C l^-1^), abbreviated with RB+OX. Carbon content was based upon literature values [23–25]. The RB concentration was close to in situ estimates of total phytoplankton carbon biomass from April through May in the southwest Baltic Sea (750 to 1500 μg C l^-1^; [26]). *Oxyrrhis marina* normally inhabits shallow water tide pools [27] but was used here since it is a valuable ecological model organism that is easy to cultivate at large quantities needed for these experiments [28]. In all tanks, abiotic and biotic parameters were measured at least once a day including temperature (9.64±0.17°C; TLog64-USB, 10-min intervals, Hygrosens, Donaueschingen, Germany), salinity (16.4±0.3; WTW cond3110 probe, Weilheim, Germany), and dissolved oxygen (9.4±0.1 mg/ml; WTW Oxi 340i probe, Weilheim, Germany) (mean±SD). Ammonium concentrations were always < 0.1 mg l^-1^ (Tetra NH_3_/NH_4_^+^ kit, Melle, Germany). Concentrations of RB and OX in each tank were measured every morning using a coulter counter (Beckman Multisizer 3 Coulter Counter, Krefeld, Germany) and adjusted by adding RB and OX as needed. Larval morphometrics, nutritional condition (RNA-DNA ratios), swimming and feeding activity, as well as digestive enzyme (trypsin) concentrations were measured each day throughout the 14-day experiment.

### Feeding and swimming activity

Each day, a total of 20 larvae was removed from each tank and carefully transferred to a 5-l opaque tank filled with 4 l of water (salinity 16.2±0.7 and 9.8±0.5°C; mean±SD). Larvae were acclimatized for 15 min then 2-d old (N1-N2), well-nourished nauplii of the calanoid copepod *Acartia tonsa* were added at a concentration of 2 ind. ml^-1^. This prey was chosen, since copepods in the *Acartia* genus are one of the dominant prey items for larval herring in the Baltic Sea [29]. Aeration was supplied to tanks which gently mixed the water. This did not appear to interfere with the ability of larvae to successfully forage for prey. Aeration was stopped during observations of swimming activity. A larva was randomly chosen and its activity was visually recorded for 2 min. This was repeated 6 times for each tank. Feeding activity was calculated as the sum of the number of aiming postures (typical s-shape) and feeding strikes performed by a larva. Pause duration was calculated as the total observation time minus the time spent moving divided by the number of stops. All measurements were done between 11.30 am and 4.00 pm with alternating observations between treatments. Larvae were allowed to forage for 4 h, after which the water level was reduced and larvae were anaesthetized with clove oil (50 ppm, 3 min) to prevent them from regurgitating or egesting prey items, and then immediately transferred to 4% buffered formalin for gut content analysis. Copepods were dissected from larval guts under a binocular microscope (Leica MZ 16, Wetzlar, Germany, 100x magnification) and counted. The *SL* of the preserved larvae was corrected for shrinkage as determined from pre- and post-preservation measurements of 20 larvae: *SL*(corrected) = 0.826*SL(preserved) + 0.844 (R^2^ = 0.896, *p* <0.001).

### Digestive capacity

Trypsin was our primary measure of digestive capacity. It is the most abundant proteolytic enzyme in marine fish larvae [30] which is present directly after hatching and has been used to monitoring short-term variability in feeding [31]. Each day, a total of 20 larvae was collected at the same time (~11.00 am) and immediately frozen at -80°C. Larvae were collected from random areas of each tank using a large bore pipette. To measure trypsin activity, individual larvae were slowly thawed on ice, dipped in de-ionized distilled water and their *SL* measured. Next, the tissue was homogenized with a micro pestle in Tris-buffer (0.1M) with CaCl_2_*H_2_O (0.02 M) (Sigma-Aldrich, Hamburg, Germany). Trypsin activity was measured spectrofluorometrically (Safas Monaco, Xenius, Monaco) in 96-well microplates (Nunc plates, VWR, Darmstadt, Germany) with Nα-benzoyl-L-arginin-4-methylcoumarinyl-7-amid as the substrate and 7-amino-4-methylcoumarin (both Bachem AG, Bubendorf, Swiss) as the fluorophore following a modified protocol from Ueberschär [32].

### Larval growth and condition

Twenty larvae were sampled each day from each tank to track changes in length, weight, and biochemical condition. After removing larvae from the tank, they were photographed (WILD M8 stereomicroscope, Olympus SZH and a Leica DC 300 camera, using Motic Images 2.0 software), dipped in de-ionized distilled water, and individually frozen at -80°C. Measurements of *SL* and yolk sac area were made using image analysis software (Image J, version 1.43u, freeware, Wayne Rasband, NIH, USA). All frozen larvae were freeze-dried (Christ Alpha 1–4 LSC, 0.200 mbar; >16 h) and weighed (Sartorius Genius SE2 microbalance, DW ± 0.1 μg).

In order to have a sufficient amount of tissue to measure nucleic acids, 2 or 3 freeze-dried larvae were combined and the tissue was homogenized with 1% sarcosil Tris-EDTA buffer (Sigma-Aldrich, Hamburg, Germany) and glass beads (0.2–2.1 mm) in a Retsch shaking mill (both Retsch, Haan, Germany). Following a modified protocol from Caldarone [33], amounts of RNA and DNA were determined spectrofluorometrically (using the aforementioned equipment) with ethidium bromide as a fluorescence-dye and restriction enzymes to eliminate the nucleic acids (as in [34]). The ratio of RNA to DNA was standardized (*sRD*) using methods outlined by Caldarone [35] using a factor of 2.4.

### Statistical Analysis

Data were tested for normality using Shapiro-Wilk tests (P = 0.05; feeding incidence data were previously arcsin transformed). Depending on the outcome, repeated measures ANOVA (RM-ANOVA) or the non-parametric alternative, the Friedman repeated measures ANOVA on ranks (Friedman-test), was performed to check for differences between replicates. For all investigated parameters, no significant differences (P>0.05) were found among the 3 replicated tanks in both treatments and hence no replicates were excluded. The daily means (n = 3) throughout the 14 days experimental period (total n = 42) were again tested for normality (Shapiro-Wilk test, P = 0.05) and checked for significant differences between the SW and RB+OX treatments (RM-ANOVA and Friedman-test, P = 0.05, df = 1). Tukey’s HSD tests were used as post-hoc tests, to control the level of the type 1 error probability. The time when 50% of the larvae had no yolk sac was calculated for all tanks with logistic regressions. All tests and regressions were executed in Sigma Plot (Systat Software, San Jose, CA).

## Results

### Swimming and Feeding Activity

#### Organismal Level

Larval swimming activity was relatively constant until 10 dph and then progressively declined in older larvae (longer pause durations, Fig 1a). No significant differences in swimming activity were observed between larvae in the presence or absence of RB+OX (Friedman-test, P = 0.76). When larvae were presented with copepods, the maximum number of feeding events occurred at 7 to 9 dph (Fig 1b) and was significantly higher in the RB+OX compared to the SW treatment (Friedman-test, P = 0.01). Copepods were found in larval gut contents of naïve larvae at 8 and 9 dph in the SW treatment and from 6 to 11 dph in the RB+OX treatment (Fig 1c). No significant differences in the incidence of feeding were found between the two treatments (Friedman-test, P = 0.10) and the percentage of larvae that contained nauplii was generally low (<15% of sampled larvae).

**Fig 1:** Mean (±S.E., n = 3 tanks) swimming activity (a), feeding activity (b), number of prey within the gut (c) and trypsin activity (d) versus age (days post hatch, dph) for yolk sac larval herring (*Clupea harengus*) reared in the absence and presence of *Rhodomonas baltica* (RB) + *Oxyrrhis marina* (OX). The black arrow indicates the age of complete yolk absorption. Significant differences between treatments were observed in feeding activity (panel b, P = 0.01, one-way repeated measures ANOVA on ranks).

#### Biochemical level

Trypsin activity ranged from 0.2 to 1.7 nmol hydrolyzed substrate MCA min^-1^ ind^-1^ and the highest values were observed at 6 dph for larvae in both treatments (Fig 1d). Although trypsin activity increased at an earlier age (4 and 5 dph) and more rapidly declined (after 7 dph) in larvae in the RB+OX treatment, no significant differences were found compared to the SW control (RM-ANOVA, P = 0.39).

### Growth

#### Organismal level

The logistic regressions predicted that 50% of the larvae had depleted their yolk by a mean (±S.E.) of 4.0(±0.2) and 3.8(±0.1) dph in the SW and RB+OX treatments, respectively. Yolk sacs were absent in all larvae ≥ 7 dph.

The larvae increased their length-at-age in both treatments until complete yolk-depletion at 6 dph (Fig 2a) and larval growth rates were essentially zero at ≥ 7 dph. Larvae in the RB+OX treatment were slightly smaller than those in the SW treatment and selection against larger individuals was greater in the RB+OX treatment (noted by the larger decrease in mean length of larvae sampled from tanks toward the end of the experiment). Weight decreased with increasing age (Fig 2b) and the decrease appeared to be most rapid from 0 to 4 dph and from 8 dph until the ‘point of no return’ at 10 dph. Between 10 and 14 dph, larvae appeared to reach a lower weight threshold. At 14 dph, the dry weight (mean ±S.E.) for larvae in SW (51.5±1.6 μg) and RB+OX (45.1±1.7 μg) treatments was half the initial weight-at-hatch (99.6±2.4 μg).

**Fig 2:** Mean (±S.E., n = 3 tanks) standard length (a), dry weight (b) and standardized RNA-DNA ratio (c) versus age (days post hatch, dph) in yolk sac larval herring (*Clupea harengus*) reared in the absence or presence of microalgae (RB) and protists (OX). Significant differences between treatments were observed in standard length (panel a, P = <0.001, one-way repeated measures ANOVA on ranks) and dry weight (panel b, P = <0.001, one-way repeated measures ANOVA). The black arrow indicates the age of complete yolk absorption. The letter ‘I’ represents the initial (common) measurement at 0 dph.

#### Biochemical level

Initial *sRD* values (0–4 dph) of yolk-sac larvae were between 3 and 5 and then steadily decreased (Fig 2c). No significant differences in the mean (±S.E.) *sRD* were observed between treatments (RM-ANOVA, P = 1.00), and at 14 dph larvae in the SW (1.32±0.09) and RB+OX (1.24±0.07) treatments had similar *sRD*.

## Discussion

During the first days after hatch, marine fish larvae rely on their yolk reserves, a phase which can last < 1 day in warm-water species to > 30 days in colder-water species [6]. Regardless of treatment, 50% of the herring larvae had depleted their yolk sac by an age of 4 dph, and no yolk remained after 7 dph. Larvae reared in the presence of microalgae and protists depleted their yolk sac marginally faster than those in the SW treatment. We speculate that this small difference was due to increased swimming activity in the presence of microalgae and protists leading to slightly higher energy (yolk) demands. In this species, the decline in the size of the yolk sac is needed before prey items such as copepod nauplii can pass through the esophagus [36] which explains the strong coupling between the decline in yolk reserves and the timing of the increase in feeding on copepods and trypsin activity. Yolk sac larvae are often capable of digesting prey using pancreatic enzymes such as trypsin prior to or at the time of first-feeding [37,38]. In our study, trypsin activity increased at 4 dph, coincident with the onset of feeding strikes on copepods. During this endogenous feeding phase, no clear distinction in growth or life span of larvae grown in the presence or absence of algae and protists was observed and larval biochemical condition (*sRD*) was most variable, likely due to the maternal transfer of RNA and differences in yolk mass [39].

At the time of first-feeding, herring larvae initially exhibit a low percentage of attacks leading to capture (40%, [40]) but quickly learn how to catch copepod nauplii and other zooplankton. Phytoplankton and protists can form an adequate prey for young, small larvae of some marine fish species while in other species larger zooplankton such as copepods are required for growth and survival [6,41]. Some protists can be more energetically costly for marine fish larvae to hunt and consume compared to larger metazoans [42] but this drawback appears to be outweighed by the positive effect of microalgae and protists on priming the digestive system which leads to precocious and intensified feeding on larger prey [18]. In their study on Atlantic cod (*Gadus morhua*), Overton and colleagues [18] observed that the ‘window of opportunity’ for feeding (when >50% feeding was observed among naïve larvae) was longest and initiated 2 days earlier in larvae reared in the presence of microalgae and dinoflagellates compared to larvae in SW controls. We found similar results for larval herring, although these results should be interpreted cautiously since the total feeding incidences we observed for herring were relatively low compared to that reported by Overton et al. [18] for Atlantic cod. When naïve herring larvae were confronted with copepods for the first time, those reared in the presence of microalgae and dinoflagellates fed more intensely and exhibited both precocious and prolonged feeding leading to a 6-day window of opportunity (6 to 11 dph) compared to only ~2 days (8 to 9 dph) of observed feeding by larvae in the SW treatment. Our results agree with recent reviews on the diets of marine fish larvae feeding which suggest that clupeids such as herrings, anchovies and sardines are amongst the taxa having the lowest (40%) median feeding incidence [6,41].

For first-feeding fish larvae, trypsin is the most important proteolytic enzyme [38]. Fish larvae deprived of larger prey tend to accumulate trypsin during the yolk-sac phase and reduce trypsin shortly after the depletion of yolk reserves [43,44]. We observed a similar trend with a peak in trypsin activity at 6 dph, coinciding with the complete depletion of yolk reserves, followed by a subsequent decline in trypsin activity. The decline was more rapid in larvae exposed to microalgae and protists (RB+OX) compared to larvae reared in SW.

At some point, fish larvae must start exogenous feeding or they will suffer starvation-induced physiological decrements leading to a ‘point of no return’ when yolks sac larvae are too weak to feed and will not survive even when prey becomes available. The ratio of nucleic acids (RNA:DNA) has been widely used as a biochemical indicator of nutritional condition (protein synthesis rate) in marine fish larvae and can rapidly decline (within 1 to 2 days) after the onset of poor feeding conditions [39,45]. Well-nourished Atlantic herring larvae are known to have *sRD* between 2 and 4 [39]. Since herring larvae were not exposed to larger prey, decrements in *sRD* and trypsin activity occurred at 60 to 80°d (10°C x 6 to 8 dph). This agrees with timing of the most rapid decline in nucleic acid ratios (60°d) observed by Peck et al. [34] for yolk sac herring reared at 8 temperatures between 5 and 19°C. Larval herring can survive about 140°days (127–153 and 110–140°days) [10,34] on endogenous (yolk) reserves. The decrements in physiological indicators starting at 60°d and the maximum life span of 140°d observed in this study indicate that algae and protists add little or no direct nutritional benefit to young larvae of this marine fish species.

## Conclusions

The role of microplankton organisms have largely been overlooked in studies examining early feeding in marine fish larvae (the ‘protozooplankton-ichthyoplankton link’, [46,47]) despite laboratory studies demonstrating that larvae pursue, attack and consume microplankton [48–50], and field studies reporting that protists can form a large portion of the gut contents of marine fish larvae [49,51]. In this study, the duration of the ‘window of opportunity’ for first-feeding was ~3-fold greater in herring larvae reared in the presence compared to the absence of phytoplankton and an heterotrophic protist. When naïve larvae were exposed to copepod nauplii, larvae reared with algae and protists attacked prey more frequently than those reared in only seawater. The presence of microalgae and dinoflagellates did not change the trajectory of growth or life span but the precocious feeding may have important implications when larger micro- and meso-zooplankton are available. Precocious feeding is likely important to growth and survival of marine fish larvae and there are potential nutritional benefits/decrements for larvae foraging on larger prey (copepods) which have consumed different types of algae and protists. Therefore, we recommend that future studies examining the role of algae and protists on yolk sac larvae include additional treatments with larger prey (copepods) and that measurements be extended into the exogenous feeding period. Furthermore, to adequately assess match-mismatch dynamics of larvae in the field, measurements of microalgae and protists should be integrated within routine monitoring programs as well as both indirect markers such as stable isotopes [51] and direct markers such as proteomics or genetic analyses of gut contents [52].
